The article "A Study of the Relationship between Blood Glucose and Serum Insulin in Acute Cerebrovascular Disease" was retracted in 2023. Reasons: unreliable results or conclusions; concerns about the data; concerns about the peer review; concerns about the citations.

# A Study of the Relationship between Blood Glucose and Serum Insulin in Acute Cerebrovascular Disease

**DOI:** 10.1155/2022/9041551

**Published:** 2022-08-01

**Authors:** Lei Zhao, Shuangling Xiu, Lina Sun, Zhijing Mu, Junling Fu

**Affiliations:** ^1^Department of Endocrinology, Xuanwu Hospital, Capital Medical University, Beijing, China; ^2^Department of Geriatrics, Capital Medical University, Beijing, China; ^3^Beijing Municipal GeriatricMedical Research Center, No. 45, Changchun Street, Xicheng District, Beijing, China

## Abstract

**Objective:**

The objective of this study was to examine the correlation between blood glucose and serum insulin with acute cerebrovascular disease.

**Methods:**

A total of 1548 patients with acute cerebrovascular illness and 364 patients with a normal physical examination who were admitted to our hospital (endocrinology department) between January 2017 and July 2020 were recruited. Patients with acute cerebrovascular illness were included in the experimental group, while healthy individuals after physical examinations were included in the control group. All patients' blood glucose and serum insulin levels were measured, and the association of blood glucose and serum insulin with acute cerebrovascular illness was investigated.

**Results:**

Acute cerebrovascular disease is associated with significantly higher blood glucose and serum insulin levels versus healthy status (*P* < 0.05). Blood glucose and serum insulin levels were observed to be significantly higher in the hemorrhagic stroke group than in the ischemic stroke or mild hemorrhagic group (*P* < 0.05). Severe ischemic strokes were associated with significantly higher blood glucose levels versus mild ischemic strokes (*P* < 0.05). There were no significant differences in serum insulin levels between the severe ischemic stroke group and the mild ischemic stroke group (*P* > 0.05).

**Conclusion:**

A rise in blood glucose and serum insulin levels is associated with the incidence and prognosis of acute cerebrovascular disease, and it is positively correlated with the severity of the acute cerebrovascular disease.

## 1. Introduction

Acute cerebrovascular disease is a common acute and critical disease in clinical medicine that causes severe damage to the brain, with high clinical mortality and disability rates [1]. Ischemic and hemorrhagic strokes are two types of acute cerebrovascular illnesses that result in coma and acute cerebrovascular events such as major cerebral infarction, vertebrobasilar artery blockage, cerebral embolism, cerebral hemorrhage, and subarachnoid hemorrhage [1]. Elderly people are more susceptible to the disease [2]. Under normal physiological conditions, the body has a complete blood coagulation system and anticoagulation and fibrinolytic systems, but if the body is in a state of reduced fibrinolysis and anticoagulation or hypercoagulation, it is prone to ischemic cerebrovascular disease and other thromboembolic diseases [3–5]. Therefore, anticoagulant drugs play an important role in acute ischemic cerebrovascular disease, among which aspirin is a common drug with antiplatelet aggregation efficacy and low cost, and is easily accepted by patients; however, its long-term application is associated with multiple adverse effects [6, 7]. Since acute ischemic cerebrovascular disease mostly occurs in middle-aged and elderly groups which generally present with different degrees of underlying pathologies such as gastric diseases, methods to reduce gastric irritation, and drug side effects and to effectively alleviate symptoms have become a hot issue of research [8, 9]. In recent years, the application value of traditional Chinese medicine (TCM) in acute ischemic cerebrovascular disease has received widespread attention, and its treatment of the disease provides unique advantages [10, 11], such as Wuchong Tongluo decoction and Buyang Huanwu decoction.

The article "A Study of the Relationship between Blood Glucose and Serum Insulin in Acute Cerebrovascular Disease" was retracted in 2023. Reasons: unreliable results or conclusions; concerns about the data; concerns about the peer review; concerns about the citations.

In recent years, the prevention and treatment of stroke patients have been a key issue in clinical practice. Stroke provokes various degrees of a stress reaction in the acute phase, and the stress response stimulates the sympathetic nerves and the hypothalamic-pituitary-adrenal axis, causing a series of aberrant alterations (diagnosed as stress hyperglycemia in such cases) [12]. With the intensive study of glucose, several studies have shown that glycemic variability is independently associated with mortality in critically ill patients. Kulkarni et al [9] retrospectively analyzed the glycemic profiles of 290,966 patients in 176 intensive care units in Australia and New Zealand from 2007 to 2016 and revealed that patients in the highest quartile of glycemic variability were at 1.43 times greater risk of death than those in the lowest quartile of glycemic variability, and after correction of the model, glycemic variability remained independently associated with hospital mortality. It is speculated that there may be an association between blood glucose levels and stroke. Research on the relationship between serum insulin and cardiovascular diseases has been conducted extensively in recent years, but there is a dearth of information on the association between serum insulin and stroke disease [13], despite a neurotransmitter or modulatory role of insulin in the central nervous system as indicated by prior research [14]. To this end, this study included 1548 patients with acute cerebrovascular disease and 364 patients with normal physical examinations, to investigate the relationship between blood glucose and serum insulin levels and acute cerebrovascular disease in order to provide a corresponding clinical reference.

The article "A Study of the Relationship between Blood Glucose and Serum Insulin in Acute Cerebrovascular Disease" was retracted in 2023. Reasons: unreliable results or conclusions; concerns about the data; concerns about the peer review; concerns about the citations.

## 2. Materials and Methods

### 2.1. General Data

A total of 1548 patients with acute cerebrovascular illness and 364 patients with a normal physical examination who were admitted to our hospital (endocrinology department) between January 2017 and July 2020 were recruited. Patients with acute cerebrovascular illness were included in the experimental group, while healthy individuals after physical examinations were included in the control group. Patients with liver and kidney diseases, as well as diabetes, were excluded, and the diagnosis was confirmed by a hematologist.

There were 78 hemorrhagic strokes and 1470 ischemic strokes in the experimental group, 51 males and 27 females in the hemorrhagic stroke group and 1029 males and 441 females in the ischemic stroke group, with a mean age of 64.68 ± 3.42 years.

In total, there were 38 cases of severe hemorrhagic stroke and 40 cases of mild hemorrhagic stroke based on their unconscious condition, the size of the lesion (the amount of blood loss, the extent of the infarction, and midline symptoms (high fever and upper gastrointestinal bleeding).

There were 402 cases of severe ischemic strokes and 627 cases of mild ischemic strokes. In addition, 364 age-matched healthy participants were included in the control group. Of these, 246 were males and 118 were females, with a mean age of 64.71 ± 3.45 years. Informed consent was obtained from patients prior to enrollment in this study. The study protocol was approved by the hospital ethics committee (ethics number: SD-ERT20170102). This experiment was performed in accordance with the Declaration of Helsinki ethical guidelines for clinical research.

### 2.2. Evaluation Criteria

5 ml of morning fasting venous blood was collected from the patients for the determination of fasting blood glucose (FBG) using the glucose oxidase peroxidase method with a radioimmunoassay kit provided by the Northern Institute of Biotechnology. The insulin was also determined by enzyme-linked immunosorbent assay (ELISA) using a Bio-RAD 550 enzyme marker and a kit from Bio-RAD, USA.

### 2.3. Grouping Methods

In accordance with the National Institutes of Health Stroke Scale (NIHSS) [15], patients were categorized according to the severity of clinical symptoms: grades 1 to 4 were classified as mild/moderate stroke, grades 5 to 15 are classified as moderate stroke, grades 15 to 20 as moderate to severe stroke, and grades 21 to 42 as severe stroke. Scores below 15 (≤15) were included in the mild group, and scores above 15 (＞15) were included in the severe group.

The article "A Study of the Relationship between Blood Glucose and Serum Insulin in Acute Cerebrovascular Disease" was retracted in 2023. Reasons: unreliable results or conclusions; concerns about the data; concerns about the peer review; concerns about the citations.

### 2.4. Statistical Methods

SPSS 22.0 software was used for data analyses. The measurement data were expressed as $\left(\bar{x}\pm s\right)$, and independent *t*-test samples were used. The enumeration data were expressed as the number of cases (%), and the *X*^2^ test was used. Statistical significance was indicated by *P* < 0.05.

## 3. Results

### 3.1. Patient Characteristics

The patient characteristics between the two groups were comparable (*P* > 0.05) (Table 1).

### 3.2. Comparison of Blood Glucose and Serum Insulin Levels between the Experimental Group and the Control Group

Acute cerebrovascular disease is associated with significantly higher blood glucose and serum insulin levels versus healthy status (*P* < 0.05) (Table 2).

### 3.3. Comparison of Blood Glucose and Serum Insulin Levels between the Hemorrhagic Stroke and the Ischemic Stroke Groups

The hemorrhagic stroke group had significantly higher blood glucose and serum insulin levels than the ischemic stroke group (*P* < 0.05) (Table 3).

### 3.4. Comparison of Blood Glucose and Serum Insulin Levels in Hemorrhagic Stroke Group

Blood glucose and serum insulin levels were considerably higher in individuals with severe hemorrhagic stroke than in patients with moderate hemorrhagic stroke (*P* < 0.05) (Table 4).

### 3.5. Comparison of Blood Glucose and Serum Insulin Levels in Ischemic Stroke Group

Severe ischemic strokes were associated with significantly higher blood glucose levels versus mild ischemic strokes (*P* < 0.05). There were no significant differences in serum insulin levels between the severe ischemic stroke group and the mild ischemic stroke group (*P* > 0.05) (Table 5).

## 4. Discussion

Acute cerebrovascular disease is one of the most common acute and critical illnesses in clinical medicine, and its major cause is senile hypertension [16]. Cerebrovascular diseases are characterized by high morbidity and mortality, and despite significant advances in clinical treatment, the 1-year survival rate of patients with cerebral hemorrhage is only 46% and the 5-year survival rate is only 29% [17]. Cerebral hemorrhage causes varying degrees of neurological dysfunction, which requires long-term hospitalization and rehabilitation and thus imposes a heavy financial burden on families and society. Therefore, the improvement of the prognosis of patients with cerebral hemorrhage has gained worldwide research attention. In recent years, it was found that hypertension is closely associated with hyperinsulinemia, insulin resistance, and glucose metabolism disorders, and insulin is an important indicator of increased blood pressure in patients [18]. Hyperglycemia is common in patients with cerebral hemorrhage, and elevated blood glucose usually indicates a poor prognosis. Van den Berghe et al. [19] found that strict glycemic control reduced mortality in patients, but some subsequent studies yielded different findings. Finfer et al. [20] found no effect of intensive insulin therapy on mortality and a significantly increased risk of severe hypoglycemia. Some studies revealed significant differences in patient prognosis even with the same average blood glucose level, and recent studies have shown that glucose variability is an independent risk factor for poor patient prognosis. Glucose variability (GV) is a nonstationary state in which blood glucose levels fluctuate between peaks and troughs. Research has suggested that glycemic variability be a novel indicator of poor glycemic control, and there are several methods to quantify glycemic variability, including mean glycemic fluctuation, coefficient of fasting glycemic variability, maximum glycemic variability, mean absolute difference in day-to-day glucose, and hypoglycemic index. However, no universally recognized gold standard is available [21]. These indices require complex calculation methods, and high economic costs are associated with limited applications.

The article "A Study of the Relationship between Blood Glucose and Serum Insulin in Acute Cerebrovascular Disease" was retracted in 2023. Reasons: unreliable results or conclusions; concerns about the data; concerns about the peer review; concerns about the citations.

According to Li Guang et al. [22], insulin resistance and compensatory hyperinsulinemia are key causes of acute cerebrovascular disease. Insulin plays a role in metabolic regulation and has a direct influence on the growth of body cells [23]. It has been speculated that insulin receptor gene mutations may weaken or even eliminate insulin's effect on regulating the growth of body cells, resulting in pathological alterations in the basement membrane of blood vessel walls, which consequently renders the microvessels brittle and increases the body weight. Acute cerebrovascular illness patients are predisposed to vascular emboli or rupture [24]. due to the pathological basis [25]. Herein, the mean age of onset is approximately 65 years, and the majority of patients have a history of hypertension. The blood glucose and serum insulin levels of the patients with hemorrhagic stroke and those with ischemic stroke were significantly higher in the experimental group than those in the control group. The increase in pancreatic islet levels may be attributed to compensatory responses or to stress reactions after disease onset. The increased insulin level in vivo is positively correlated with the severity of acute cerebrovascular disease [26], indicating that the higher the insulin level in the patient, the worse the prognosis of the patient [27].

The article "A Study of the Relationship between Blood Glucose and Serum Insulin in Acute Cerebrovascular Disease" was retracted in 2023. Reasons: unreliable results or conclusions; concerns about the data; concerns about the peer review; concerns about the citations.

The increase of intracranial pressure in cases with acute cerebrovascular illness or lesions that damage the midline of the brain may impact the hypothalamus directly or indirectly and prompt the pituitary gland to produce and release hormones. Some cell breakdown products such as serotonin may trigger vasospasm in the body during cranial hemorrhage, exacerbating hypoxia, and ischemia of the hypothalamus and pituitary gland, resulting in the endocrine condition [28]. Zhang Tianli et al. [29] suggested that, in patients with acute cerebrovascular disease, the larger the lesion, the greater the cerebral edema and mass effect in the body, which also causes the displacement of body tissues, including the hypothalamus and pituitary glands [30].

In the present study, blood glucose and serum insulin levels were substantially higher in the group with severe hemorrhagic stroke than in the group with moderate hemorrhage. Blood insulin levels of patients with severe ischemic stroke and moderate ischemic stroke were significantly higher than those of individuals with mild ischemic stroke. The comparison of serum insulin levels in the ischemic stroke group did not show statistical significance, which is mostly attributed to the limited number of cases, and its relevance requires more data for verification [31].

Relevant clinical studies have demonstrated that hyperglycemia could exacerbate brain damage in patients with acute cerebrovascular disease.

1. Due to the elevated blood glucose concentration in the patient, the ATP supply in the patient's body is insufficient under ischemia and hypoxia, resulting in a large amount of glucose via anaerobic glycolysis. This produces a severe lactate buildup that inhibits mitochondrial energy production in the patient's body, ultimately depleting the patient's body's energy supply and thus, exacerbating their brain injury [32];
2. Changes in local cerebral blood flow in patients: hyperglycemia could increase the viscosity of the patient's blood and lead to a decrease in the deformability of red blood cells, thereby preventing the red blood cells from establishing an effective collateral circulation during cerebral infarction and resulting in reflex vasospasm in the body, which will aggravate cerebral ischemia, brain tissue edema, and enlarged necrotic areas in the brain, thereby increasing intracranial pressure [33];
3. Intracellular Ca2^+^ overload: the water and sodium retention, along with free radical damage in the body will aggravate the destruction of the body's inner membrane structure, thereby accelerating the necrosis process of the individual cells of the patient [34].

The article "A Study of the Relationship between Blood Glucose and Serum Insulin in Acute Cerebrovascular Disease" was retracted in 2023. Reasons: unreliable results or conclusions; concerns about the data; concerns about the peer review; concerns about the citations.

There are some limitations to this study. First, this study was conducted in a single center with a small sample size. Second, the possibility that differences in patient populations may have an impact on neurological outcomes cannot be excluded. Comorbidities such as diabetes mellitus were not examined herein. Third, blood glucose was collected based on clinical need, and data were not collected at equal intervals and frequencies. Fourth, due to the small sample size, no correction could be performed in the subgroup analysis. Future studies with large samples may correct patients for subgroup analysis to ensure the reliability of the results.

A rise in blood glucose and serum insulin levels is associated with the incidence and prognosis of acute cerebrovascular disease and is positively correlated with the severity of the acute cerebrovascular disease.

## Figures and Tables

**Table 1:** Patient characteristics [*n*(%)].

	Experimental group (*n* = 1548)	Control group (*n* = 364)	*t*/*x*^2^	*P*
Gender			0.005	＞0.05
Male	1080	246		
Female	468	118		
Age (years)	$\left(\bar{x}\pm s\right)$	$\left(\bar{x}\pm s\right)$		
Mean age (years)	64.68 ± 3.42	64.71 ± 3.45	−0.177	＞0.05
Pathological type				
Hemorrhagic stroke	78			
Ischemic stroke	1470			
Order of severity				
Mildly hemorrhagic	40			
Severely hemorrhagic	38			
Mild ischemia	402			
Severe ischemia	627			

**Table 2:** Comparison of blood glucose and serum insulin levels between experimental and control groups $\left(\bar{x}\pm s\right)$.

Group	Cases	Blood glucose (mol/L)	Serum insulin (U/L)
Experimental group	1548	8.16 ± 6.28	25.78 ± 9.89
Control group	364	5.85 ± 0.83	11.45 ± 4.37
*t*	—	8.04	29.543
*P*	—	＜0.05	＜0.05

**Table 3:** Comparison of blood glucose and serum insulin levels between the hemorrhagic stroke and the ischemic stroke groups $\left(\bar{x}\pm s\right)$.

Group	Cases	Blood glucose (mol/L)	Serum insulin (U/L)
Hemorrhaging stroke group	78	10.77 ± 7.15	34.48 ± 9.47
Ischemic stroke group	1470	7.80 ± 6.43	21.88 ± 9.86
*t*	—	8.34	26.724
*P*	—	＜0.05	＜0.05

**Table 4:** Comparison of blood glucose and serum insulin levels in hemorrhagic stroke group $\left(\bar{x}\pm s\right)$.

Group	Cases	Blood glucose (mol/L)	Serum insulin (U/L)
Mild hemorrhagic stroke group	40	9.88 ± 5.27	26.11 ± 11.13
Severe hemorrhagic stroke group	38	11.85 ± 8.30	41.68 ± 7.95
*t*	—	−4.24	26.72
*P*	—	＜0.05	＜0.05

**Table 5:** Comparison of blood glucose and serum insulin levels in ischemic stroke group $\left(\bar{x}\pm s\right)$.

Group	Cases	Blood glucose (mol/L)	Serum insulin (U/L)
Mild ischemic stroke group	402	6.51 ± 3.22	21.68 ± 9.72
Severe ischemic stroke group	627	13.73 ± 12.92	22.58 ± 11.78
*t*	—	−12.304	−1.045
*P*	—	＜0.05	＞0.05

The article "A Study of the Relationship between Blood Glucose and Serum Insulin in Acute Cerebrovascular Disease" was retracted in 2023. Reasons: unreliable results or conclusions; concerns about the data; concerns about the peer review; concerns about the citations.

## Data Availability

No data were used to support this study.
